# Eliminating Data Duplication in CQA Platforms Using Deep Neural Model

**DOI:** 10.1155/2022/2067449

**Published:** 2022-08-25

**Authors:** Seema Rani, Avadhesh Kumar, Naresh Kumar

**Affiliations:** School of Computing Science & Engineering Galgotias University, Greater Noida, Uttar Pradesh, India

## Abstract

Primary research to detect duplicate question pairs within community-based question answering systems is based on datasets made of English questions only. This research put forward a solution to the problem of duplicate question detection by matching semantically identical questions in transliterated bilingual data. Deep learning has been implemented to analyze informal languages like Hinglish which is a bilingual mix of Hindi and English on Community Question Answering (CQA) platforms to identify duplicacy in questions. The proposed model works in two sequential modules. First module is a language transliteration module which converts input questions into a mono-language text. The next module takes the transliterated text where a hybrid deep learning model which is implemented using multiple layers is used to detect duplicate questions in the mono-lingual data. The similarity between the question pairs is done utilizing this hybrid model combining a Siamese neural network with identical capsule network as the subnetworks and a decision tree classifier. Manhattan distance function is used with the Siamese network for computing the similarity between questions. The proposed model has been validated on 150 pairs of questions which were scrapped from various social media platforms, such as Tripadvisor and Quora which achieves accuracy of 87.0885% and AUC-ROC value of 0.86.

## 1. Introduction

With the wireless access to the Internet becoming pervasive, recent years have seen an incessant advancement in Web usage with new user-centric applications and media-rich services. Social media has become an integral and indispensable part of our lives. Social networks make sharing of information, communication, and collaboration straightforward and opportune. The social media websites have grown significantly popular over the past decade as open-source platforms for information and knowledge sharing. Social media has become a primary source of the big data. Formally, big social data are the voluminous and varied data with high-velocity that is generated from technology-mediated social interactions and actions in online realm, and which can be scrapped and mined to comprehend social interactions and behavior. Undeniably, big data and social business intelligence are the key components for reaping full ROI.

Social media has been developing momentously and has changed the dynamics of the sharing and learning ecosystem. Social media news feeds and question answering sites are increasingly becoming popular valuable resource material for enriching knowledge base. The emerging role of social media in teaching-learning process cannot be ignored. Community Question Answering (CQA) [1] as a crowd-sourced service has emerged as a collective intelligence social system which facilitates participation of volunteers to express their knowledge and clear their uncertainties regarding some topics. It allows collaborative user participation where some users ask questions and the others provide answers to them. The number of participating users and the volume of questions and answers of different varieties characterize the popularity of CQAs.

Though these sites have high informational value while on the other hand in order to filter out the relevant information in the form of best answers, or answers by experts for reliable information and user satisfaction, it requires time and labor. Some of the challenges associated with these platforms include ambiguity in user preference, duplicity in the questions, fuzziness, and imprecision among the huge and speckled answers [2]. The regular influx of new questions and getting answers to questions requires detecting semantic equivalence of questions. The problem of detecting semantic equivalence of multiple sentences is prevalent in natural language processing tasks. The problem further extends if there exists multilingual text or text using mash-up of varied languages like Hinglish.

Numerous CQA sites provide forum which contains answers to existing questions, and users are recommended to search the forum before posting their questions but it may not work as a same question may be rephrased in different ways and languages. There exist duplicate detection policies in some platforms, but these are limited to exact duplicate questions as well as near-exact duplicates. However, some of the challenges associated with analyzing questions for semantic equivalence detection are as follows:

- There are multiple ways to rephrase a same question
- There may exist same solution to different questions
- A question may be phrased in a mash-up of two languages
- Merging of question threads is required after duplicate questions have been answered
- There exist volumes of historical questions

The first two cases define the issue where questions are in an asymmetrical domain. The examples in Figure 1 expound the first three cases.

Maximum number of primary studies on duplicate question detection deals with English-only CQAs. The cultural diversities, country-specific trending topics—hash-tags on social media, and availability of native language keyboards add to the user-generated content in multiple languages contributing the linguistic challenges [3]. Linguistic anglicization of a language which is defined as to make a language sound or appear in English is a commonly observed phenomenon where one language/script word is transcribed into a source language so as to preserve source phonetics. For example, the question “Kya roz exercise krna zruri hai?” is a transliterated on the basis of pronunciation of bilingual mix of Hindi and English called Hinglish. The transliteration is not based on meaning. Instinctively, the question semantically becomes similar to the mono-lingual English question “Is daily exercise important?”

With recent upsurge in transliterated bilingual posts on CQAs which are restricted by their mono-lingual abilities and lack of collective part-of-speech taggers, it is essential to explore techniques that extend the cognitive capabilities of machines to interpret, comprehend, and learn features for semantic matching in multilingual (bilingual/trilingual) data. This research put forward a solution to resolve the problem of detection of semantic equivalent questions for duplicate detection in transliterated bilingual data. The proposed model examines the semantic similarity for input questions of varied languages using deep learning-based Siamese neural networks. In recent studies, evidences exist where deep learning techniques are achieving advanced results on specific natural language processing-based problems as these possess hierarchical learning capabilities and are capable of generalizations [4, 5]. Siamese neural network is a deep learning-based technique comprising more than one identical subnetworks having same configuration (parameters and weights) [2, 6, 7]. The subnetworks of Siamese neural network are built on various categories of neural networks including convolutional neural networks and capsule networks. Semantic matching using Siamese neural network is performed by transforming the input sentences at each subnetwork into vectors and using a Manhattan distance function.

Thus, the proposed framework comprises two submodules first being the language transformation module and the second being the semantic matching module. As a first step, the input text containing questions is converted into a mono-language using language transliteration and translation tools. Further, a hybrid deep learning model is used for identification of duplicate questions in mono-language. Similarity detection between question pairs is carried out using a hybrid model using Siamese neural network combining with decision tree (DT) classifier. The Siamese neural network is built up of two identical capsule networks [8, 9] with same configuration, and Manhattan function is used as a distance measure for evaluating the similarity among questions. Further, DT classifier is used at the output layer which produces whether a question pair is duplicate or not. A dataset of 150 question pairs has been used to validate the proposed. The questions have been scrapped from multiple CQA forums like Tripadvisor and Quora.

The manuscript is structured as follows: Section 2 explores the literature review related to the domain of the study, Section 3 explains the proposed methodology, Section 4 presents the results, and Section 5 concludes the study.

## 2. Related Work

The growing number of Internet users in around interactive networking sites has increased researchers' interest to intelligently mine the user-generated online content. The utilization of machine learning and deep learning techniques for providing solutions to various problems of natural language processing tasks with user-generated online data has been evident to give accurate results. The potential of analyzing user-generated online content with intelligent data analysis techniques has provided solutions to various natural language processing problems which include sentiment analysis [4, 10], sarcasm detection [3, 11], rumor detection [12, 13], etc.

The large data generated by users each day on CQAs make it necessary to filter relevant data by discarding duplicate data. First step to achieve this is to analyze the data in order to detect duplicate questions by semantically matching the text. Multiple researchers have attempted to detect semantically equivalent sentences. Dey et al. [14] employed support vector machine (SVM) for identification of semantically equality in blogs using the SemEval-2015 dataset. Siamese neural network which encodes two input sentences encoding those using same neural networks has been used recently to detect semantic equivalence of sentences and has shown accurate results [6, 7, 15]. In studies [16, 17], dataset of Quora has been analyzed for duplicate detection utilizing various connection networks. Rodrigues et al. [18] present performances of efficient experiments on detection of duplicity in questions using the established approaches and proposing a novel method. Chen et al. [19] attempt to solve duplicate question detection problem on Quora by a feature engineering and a neural-network-based model. Zhang et al. [20] propose a novel model named DupPredictor in order to recognize possible duplicates of an original question on stack overflow. In another study [21], the authors propose a model utilizing classification algorithms for duplicate question detection on stack overflow. They named their model as Dupe. Reproduction of DupPredictor as DupPredictorRep and Dupe as DupeRep has also been executed by Silva et al. [22] conducting advanced experiments. The use of Siamese neural network for resolving problem of duplicacy in CQA has also been seen in recent studies. Kumar [2] proposes a Siamese neural network model with attention-based bidirectional long short-term memory as subnetworks for detection of duplicate questions in medical CQAs.

The existing studies in the domain of matching of duplicate questions are done with English questions only as the current CQA forums provide facilities to post in one language only, mainly English only. Existing studies deal with question only in English language and deal with other language questions as noise. In a recent study [23], authors explored a code-mixed Q&A platform for Indian languages including Tamil and Hindi, their mash-up with English.

## 3. The Proposed Siamese Capsule Network with Manhattan Similarity

The proposed model comprises two modules. First one is the language transformation module, and second one is the semantic matching module (Figure 2).

The following sections describe the working of each module of the proposed framework in detail.

### 3.1. Language Transformation

The tokens of Hinglish are decoded in this module using transliteration into Hindi, and subsequently the Hindi words into English language are translated. “Transliteration is the process of converting a text in one language to text in another language on the basis of its pronunciation (maintaining it to greatest possible extent) without the change in grammar” [24]. Transliteration is different from translation in a manner that it is based on the pronunciation in the aimed language, while translation is based on the meaning in the target language (Figure 3). For instance, for the Hindi phrase “किस उम्र में बच्चों को इंटरनेट यूज़ करने देना चाहिए?” its translation in English would be “At what age should children be allowed to use the Internet?” and “Kis umar mein bachon ko Internet use karne dena chahiye?” is the transliterated Hindi. In this work, the Google Transliteration–Translator toolkit (Google Input Tools: https://www.google.co.in/inputtools/try/) has been used for the task of transliteration of code-mixed text into English in this module. The purpose of using a two-step transformation is imperative to capture the right textual interpretation. Using the Google Translate independently may not always output the correct meaning (Figure 3).

The correct interpretation for the example in Figure 3 would be “Should chocolate be eaten in depression?” and therefore, to improve the meaningfulness of transliterated text, the language transformation follows these steps (Figure 4):

- Word-level transliteration is done to convert Hinglish text to Hindi
- Sentence-level translation is done to translate Hindi to English

This translated English question is then input to the Siamese network to match the semantics with the English-only input. The next section discusses the details about the semantic matching module.

### 3.2. Semantic Matching

Semantic matching of question pairs is done using a Siamese capsule network. Siamese neural network is made up of two neural networks of same configuration (parameters and weights) each taking different inputs. An energy function which compares feature representations of highest level on each side of the network by assessing a metric is used to join these two neural networks. Similarity among the two inputs (questions) is evaluated by transforming the inputs into representation vectors and using a distance function. We use Manhattan distance function for calculation of the similarity between all question pairs. The vector representations from the encoder are fed to the DT model together with their distance for binary classification.

#### 3.2.1. Input Layer

This layer accepts questions as inputs into each subnetwork of the Siamese model. The question pair is further passed to the embedding layer.

#### 3.2.2. Embedding Layer

In this study, GloVe [25] which is a count-based model is used for word embeddings in the embedding layer. In this layer, the input textual format is converted into vector table of words using GloVe. A real-valued vector of words is built as pretrained word embedding. Each question's embedding matrix is sent into the next layer.

#### 3.2.3. Encoding Layer: Siamese Capsule Network

In this layer, the output of GloVe (word matrix) is converted into a one-dimensional feature vector. In this work, the encoding layer is employed using capsule network [8, 9]. The capsule network is composed of capsules which are groups of neurons. These groups are locally invariant groups with the capability of recognizing visual entities and encoding their features into vectors [26]. A capsule network comprises three layers including convolutional layer, primary capsule layer, and class capsule layer. Each layer provides a unique functionality given in following sections.

*(1) Convolutional Layer*. The vector representation of the text is provided to the filtration layer of the convolution having 128 filters of 8 size each, after applying a randomized function over the vectors. These filtered feature vectors are given as an input to a nonlinear function that acts as a linear function and uses stochastic gradient descent to train the model and to avoid the saturation problem of other activation functions. The rectified linear activation function has used the third layer of CNN, so named as ReLU activation layer. In each convolutional layer, the output from *i*th feature map, given by *y*_*i*_^*l*^, after the convolution operator is calculated as given in

(1) $$\begin{array}{c} y_{i}^{l}=b_{i}^{l}+\sum_{j=i}^{m}f_{i,j}^{l}*y_{j}^{l-1}, \end{array}$$

where *l* is the layer having *m* filters, *f*_*i*,*j*_^*l*^ is the convolution filter, *y*_*j*_^*l*−1^ is the output obtained from the previous layer, and *b*_*i*_^*l*^ denotes the bias matrix.

*(2) Primary Capsule Layer*. The scalar inputs from the lower convolution layers are passed onto the first capsule layer. Here, these inputs are converted into vector outputs which are called capsules. Capsules intend to preserve the instantiate parameters including the syntactic or semantic representations of word and their local order. The features produced by the lower convolutional layers are further produced as combinations of features grouped into capsules in this layer, and a routing algorithm is implemented for communications with the upper layer. A capsule in the upper layer is activated if numerous lower layer capsules vote for that capsule. Results from lower level capsules are broadcasted to that activated upper level capsule. A cluster of capsules coming from lower layer is created at this activated capsule and a high probability of observation that an entity is present and a high-dimensional pose is produced as an output at the higher-level capsule.

For semantic matching of two sentences, it is difficult to say that two sentences are different because the order of the sentences is different. Hence, in this work we use the capsule network with routing algorithm as static routing algorithm.

Let *u*_*i*_ be the output of a single capsule, then the equation for static routing is as follows:

(2) $$\begin{array}{c} s_{j}=\sum_{i}W_{ij}u_{i}. \end{array}$$

Here, capsule “*i*” is in the primary capsule layer which is the current layer, capsule “*j*” is a capsule in the higher level, and *W*_*ij*_ is translation matrix.

*v*_*j*_ is the output vector limited to [0, 1] as the result of applying squashing function to *s*_*j*_ as given below:

(3) $$\begin{array}{c} v_{j}=\frac{{\left|s_{j}\right|}^{2}}{1+{\left|s_{j}\right|}^{2}}\;\frac{s_{j}}{\left|s_{j}\right|}. \end{array}$$

*(3) Class Capsule Layer*. This layer is the capsule network's final capsule layer which takes inputs from the lower layer through a static routing algorithm, also called the routing by agreement.

*(4) Similarity Measure*. This study utilizes the exponential function on the negative value of distance measured by Manhattan distance function to find the similarity distance between the vector representations. This is represented in

(4) $$\begin{array}{c} \text{exp}\left(-\left\|v1–v2\right\|\right)\in \left[0,1\right], \end{array}$$

where *v*_1_ and *v*_2_ represent the outputs of subnetworks.

#### 3.2.4. Output Layer

Decision tree (DT) classifier is implemented at the output layer to make the final prediction. DT is a tree-based model which comprises a root, branches, and leaf nodes where the dataset information is broken down into smaller subsets till an associated decision tree is built. The input attributes are allied with the nonleaf nodes, and the classes are represented by the leaf nodes. The output of Siamese network is sent to DT classifier which models the interaction between the two questions. The output of Siamese encoder is fed to DT generating a hybrid Siamese neural network and DT classifier which models the interaction between the two questions. The concatenation of the representations of questions with their distance, *c* = [*f*(*q*1); *f*(*q*2); *d*(*q*1, *q*2)], is given as input to DT, and the probability of a match between them is produced as output.

## 4. Results

Section 4.1 discusses the dataset used in this study to validate the proposed model, and Section 4.2 discusses performance of the proposed hybrid model.  Section 4.3 describes the performance analysis of various question types, and Section 4.4 compares the Manhattan distance measure with various other distance measures. Lastly, Section 4.5 shows the comparison of the accuracy of the proposed hybrid model with different variants of Siamese subnetworks.

### 4.1. Dataset

The data are prepared by extracting 150 pairs of questions from CQA forums including Tripadvisor and Quora. It consists of pairs of questions each having one question in English, and one is in Hinglish script. The dataset is labeled with “duplicate” and “nonduplicate” for each question pair.  Table 1 presents a sample snapshot of the data.

### 4.2. Performance of Proposed Framework

The performance of the proposed Manhattan hybrid Siamese neural network model with DT classifier for similarity matching is evaluated in terms of accuracy and AUC-ROC. “Accuracy is defined as the proportion of correct predictions to the total number of predictions.” “ROC curve (receiver operating characteristic curve) is a graph measuring the performance of a classification model by plotting true-positive rate against false-positive rate.” “AUC stands for area under the ROC curve which measures the entire two-dimensional area underneath the entire ROC curve.” Optimal selection of parameters is imperative to achieve superlative performance results. The hyper-parameters are tuned using the validation data in order to obtain accurate results. GloVe is implemented with dimensions of 300 and a batch size of 60 and 0.5 drop-out.

The confusion matrix and ROC graph plots for the same are given (Figures 5 and 6). The confusion matrix is a plot of true positive, false positive, false negative, and true negative. The model attains an accuracy of 87.0885%. The results show that it is predicting accurate results in identifying correct and incorrect answers. The value of the precision column indicates low false-positive rate. It does not identify wrong answers as correct answers. Higher recall value suggests that our system makes less mistakes in classifying the answers of a question. It can correctly predict that is the answer right or wrong. Because the recall value is high, there are fewer forecasts when the actual answer is true but the system predicted incorrectly.

Finally, *F*1 score is basically the average of two quantities that is the precision and the recall in which we consider the false positives and the false negatives. Higher *F*1 score establishes that our system makes less mistakes.

### 4.3. Performance on Different Question Types

The accuracy of the proposed hybrid framework has been evaluated for various question types such as “what,” “who,” “why,” “when,” “where,” “which,” “are,” “is,” “should,” and “how” using the exact match measure which is represented in Figure 7.

It can be seen that the best predictions can be made for questions of type “when.” The next best predictions are made for the questions beginning with “who” and “how,” whereas least accuracy was achieved with the “why”-type questions.

### 4.4. Comparison of Various Similarity Measures

The performance of the model using the Manhattan distance has been compared with the models using Euclidean and cosine distances as similarity measures. The results are shown in Figure 8.

The model using Manhattan distance performs best, and the model using cosine distance gives the worst performance.

### 4.5. Assessment of Other Subnetworks

The accuracy of the proposed hybrid model has also been compared with Siamese models having different neural network architectures at the subnetworks. The other models which have been evaluated for the detection of duplicate question pairs in transliterated bilingual data are as follows:

- Siamese MLP network
- Siamese LSTM network
- Siamese CNN

Manhattan distance for similarity measure and the same dataset has been used in all the models. The comparative performances are given in Figure 9 where the *y*-axis denotes the accuracy percentage plotted for each model on the *x*-axis.

As seen in the figure, the proposed methodology utilizing hybrid Siamese capsule network with DT classifier and Manhattan similarity outperforms the other Siamese neural network models' semantic similarity matching in transliterated bilingual data.

## 5. Conclusion

The large volume big data generated through the communications through social networks makes it imperative analysis for data-driven decision making. But adversarial IR (targeting, probing, spam traps), multilingual, and duplicate content are the key issues that challenge the performance of a typical CQA. This study proposes a hybrid model combining a Siamese neural network with capsule network as a subnetwork and a decision tree classifier to detect duplicate pairs of questions. For the problem of semantic question matching for duplicate detection in transliterated bilingual data on CQA, the input questions are transformed into a single language using language transliteration and translation tools. Manhattan distance similarity measure is used with the deep learning model for similarity match between the question pairs. The proposed hybrid model achieves an accuracy of 87.0885%. The limitation of the work includes lack of benchmark datasets. In future, we intend to build a language-independent framework for identifying semantic similarity which could comprehend duplicates in bilingual or trilingual data. The model can also be trained and tested for visual question answering. Further studies on types of mash-up including code-mix and code-switch input types can also be done.

## Figures and Tables

**Figure 1:** Challenges in CQAs.

**Figure 2:** The proposed model.

**Figure 3:** Sample independent use of Google translation.

**Figure 4:** Transliteration: Hinglish to Hindi and translation: Hindi to English.

**Figure 5:** Confusion matrix.

**Figure 6:** ROC curve.

**Figure 7:** Accuracy obtained on different question types.

**Figure 8:** Comparative performance using varied distance functions.

**Figure 9:** Performance of various subnetworks.

**Table 1:** Snapshot of dataset.

English question	Hinglish question	Is duplicate?
Which animal would you like to pet	Aapka favorite jaanvar kya hai	N
Are you satisfied with your life	Kya aap jeevan m aur paise kamana chahte hai	N
What are the benefits of eating mango	Mango khaane k kya faayde hai	Y
How to follow your passion	Apne passion ko kaise sakar kare	Y
How to lose belly fat	Kamar k aas paas ka fat kaise ghataye	Y
Should we drink green tea	Kaunse brand ki green tea peeni chaiye	N
How much does a road trip from LA to Vegas cost	Las Vegas se LA jaane ke liye kya options hain	N
Is daily exercise important	Kya daily exercise krna zruri hai	Y
How to open WhatsApp Web on desktop	Desktop pe WhatsApp kaise use karte sakte hain	Y
Which places to visit in Mumbai	Mumbai mein best beach kaunsa hai	N

## Data Availability

Data will be made available on request.
